# Practice and Reflection on Piano Teaching Reform of Music Major in Colleges and Universities under Diversified Environment

**DOI:** 10.1155/2022/9688655

**Published:** 2022-07-30

**Authors:** Ya Huang

**Affiliations:** Shijiazhuang University, Shijiazhuang 050035, Hebei, China

## Abstract

In order to further promote the innovative development of piano teaching of music major in colleges and universities under a diversified environment, we explore a modern piano teaching reform with distinctive innovative characteristics and strengthen the work needs of colleges and universities for the cultivation of comprehensive, practical, and high-quality piano talents. This study deeply understands the current piano learning, curriculum teaching, and innovative practice of music majors in colleges and universities in the form of questionnaire and interview. On this basis, based on the summary of piano teaching methods, this paper puts forward a piano teaching curriculum system based on innovative development, hoping to provide reference and suggestions for the innovation, reform, and development of piano teaching of music majors in colleges and universities.

## 1. Introduction

The development of the network and the advent of the information age have brought about not only great changes in various fields but also have caused changes and development in various fields. Especially under the influence of the Internet, there are more and more media tools in the diversified environment and even have penetrated people's life and learning. In the diversified environment, the Internet is also a modern teaching carrier. In the process of pursuing the reform of the teaching system, the intervention of the network and the integration of multimedia have also been penetrated and optimized to varying degrees. Network education in a diversified environment has played a positive role in the process of music teaching reform, has a positive impact on changing the traditional teaching methods and innovating the curriculum teaching system, and has also promoted the diversified development of music teaching in modern colleges and universities. At the same time, the teaching methods of piano courses in colleges and universities show a diversified development trend. Based on this, this study is based on a diversified teaching environment to explore the distinctive piano teaching reform, as shown in Figure 1.

## 2. Literature Review

As the use of digital technology continues to improve and the information age emerges, piano lessons are gradually entering a new era of network development. In the early 1990s, Europe and the United States were encouraged to use teaching materials, traditional teaching technologies, and a variety of teaching methods. Thus, it played an important role in supporting education reform in Europe and the United States after the new century. As a result, many European countries have enacted the law, opening up new opportunities for online learning around the world [1].

As music education develops and improves, more and more attention is paid to the quality of piano instruction. Many top teachers and music therapists have researched this topic and published numerous studies on its accomplishments. Currently, the research done in this field is focused on the following points.

Research on improving piano learning: Some scholars temporarily link musicians and their work to produce in-depth research on the development of music in China and piano training (Pател, ES). It is believed that piano lessons began in China after the introduction of piano in China. After hundreds of years of research and practice, the Chinese piano industry has formed a large group, trained many musicians, and made more and more competition in Chinese piano learning. Through the constant efforts of piano teachers, Chinese piano art has developed rapidly, promoting the development of Chinese music culture and art; Juan studied the development of piano lessons at various levels and levels of Chinese piano on piano instruction in professional colleges and had developed optional piano instruction manuals and instruction manuals for piano in social studies [2].

Research on piano teaching of music education major in colleges and universities: Some scholars put forward opinions and suggestions on how to improve piano education in normal universities, and analyzed the phenomenon of reform in detail; Ellawala analyzed the current teaching situation of piano playing ability, sight reading ability, improvisation accompaniment ability, and cooperation ability and gave suggestions on how to improve these abilities [3].

Research on the teaching content and teaching purpose of piano: Some scholars take Yanbian University and some professional art colleges and normal universities in China as the research center to study the piano teaching content of these schools, and make a comparative study with the method of comparison; Efremova N. did systematic research and analysis from three aspects: the teaching purpose, teaching content, and teaching method of piano course for normal university [4]. Sun summarized his music experience in six contemporary music fields: piano art, comparative music, ethnomusicology, music education, music philosophy, and music aesthetics [5]; Wa studies the talent training mode from the perspective of higher music education, systematically combs and analyzes the history of the emergence and development of music education at home and abroad, provides examples and ideas for the creation of higher music education training mode, and puts forward the strategy of constructing the talent training mode of higher art education conducive to people's comprehensive development and social progress through the analysis of typical cases of music education at home and abroad [6].

## 3. Investigation on the Current Situation of Piano Teaching of Music Major in Colleges and Universities

### 3.1. Questionnaire Survey

Combined with the research theme, this survey takes four colleges and universities in a city (art colleges, normal colleges, comprehensive universities, and higher vocational colleges) as the research object. We fully understand the basic situation and class situation of the students studying piano lessons in the school, interview the students majoring in music education who are reading or have graduated, and then continue to conduct sampling survey, starting from the basic situation of the students, to the students' piano learning and the school's piano teaching, including teaching resources, teaching contents, teaching forms, assessment methods, etc.

A total of 31 questions and 30 statistical tables were set in this questionnaire. The method of sampling survey was adopted to conduct an anonymous questionnaire survey on college students. The questionnaire understands college students' views on piano teaching in their school from four aspects.

Implementation: from September 2021 to December 2021, 200 questionnaires were distributed to students majoring in music education in these four colleges and universities, and 196 questionnaires were recovered, with a recovery rate of 98%.

### 3.2. Investigation

#### 3.2.1. Basic Information of Students

The survey on the basic situation of students includes four questions, including the place of origin of students, piano learning at the time of admission, piano playing level, and spectrum recognition.

It can be seen from Table 1 that students from cities account for 22%, township students account for 44%, and rural students account for 34%. At the same time, it also reflects that the current development of piano education in this area is not universal enough, and the development of urban piano basic education is better than that in rural areas.

As can be seen from Table 2, not many students have been studying piano before the age of 10, accounting for only 13% of the total number of respondents. Some students have systematically studied the piano for 1–3 years at the time of admission. About 44% of the students only came into contact with the piano before the art examination. Most of them were admitted to the current school through surprise learning before the art examination. They have almost no piano foundation, and the piano repertoire they contact is also very limited. There are only one or two pieces during the examination, and 14% of the students chose almost no piano [7].

It can be seen from Table 3 that with the improvement in piano playing degree, the difficulty of playing repertoire increases and the number of people decreases, which also reflects the difficulty in the piano learning process and the uneven piano level of music teaching students in colleges and universities in the city [8].

#### 3.2.2. Investigation of Students' Piano Learning

There are four questions in the investigation of students' piano learning, which are asked and investigated according to the students' weekly piano practice time, difficulties encountered in piano learning, concerns during piano practice, whether to consult data before playing, as well as the contact with works, track sources, accompaniment ability, and accompaniment learning [9].

The students' enthusiasm and attention to piano courses can be understood from Table 4 as follows: 32% of students practice piano for only 2–4 hours a week, 43% of students practice piano for 5–10 hours a week, and 25% of students practice piano for more than 10 hours a week.

The students' attitudes toward learning piano and practicing piano in ordinary times can be understood from Table 5. 14% of students pay attention to whether they can return lessons, 32% of students pay more attention to whether they can play completely, 29% of students pay attention to whether they master technical essentials, and only 25% of students pay attention to whether they have musical treatment when practicing piano [10].

As can be seen from Table 6, only about 11% of students never consult relevant materials before playing piano works.

In addition to piano solo works, 11% of students are often exposed to some cooperative works, 48% of students are occasionally exposed to some cooperative works, and 41% of students are not exposed to any cooperative works according to Table 7 [11].

From the questions in Table 8, the students' ability of improvisation accompaniment is investigated. Only 8% of the students can play improvisation accompaniment well, 56% of the students think they can play a little through practice, and 36% of the students cannot play improvisation accompaniment at all [12].

From Table 9, it can be seen that from the survey of interest in piano impromptu accompaniment course, 90% of the students are more interested in this course and only 10% of the students are not interested or indifferent to this course [13].

#### 3.2.3. Piano Teaching in Colleges and Universities

The teaching resources: from Tables 10 and 11, 39% of the students think that the school provides enough pianos for practice, and 61% of the students think that the school has less pianos, which cannot meet the needs of piano practice. 47% of the students think that the school library has enough literature and audio-visual materials, and 53% of the students think that the school library does not have enough literature and audio-visual materials [14]. The number of documents and audio-visual materials in the school is not enough to meet the needs of students.

The teaching content: it can be seen from Tables 12 and 13 that most teachers often or occasionally involve relevant music-theoretical knowledge and explore daily piano practice methods in the process of piano teaching. Only about 10% of teachers never involve relevant music theory knowledge in the process of piano teaching, and about 16% of teachers do not discuss daily piano practice methods with students in the process of piano teaching [15].

The statistics in Tables 14 and 15 show that in piano lessons, most teachers focus on piano performance, and a few teachers focus on piano performance, the ability to participate in piano lessons, and only music instructions.

As Table 16 shows, teachers use a variety of techniques to teach students piano instruction, including teaching, modeling, and practice [16, 17].

The teaching method: it can be seen from Tables 17 and 18 that 40% of students take individual classes, 42% take group classes, and 18% take collective classes. 46% of school academics often participate in lectures, concerts, and other academic exchange activities, 45% of students occasionally participate in these academic exchange activities, and 9% of students never participate in academic exchange activities [18].

#### 3.2.4. Investigation on Students' Practice

According to the results of Tables 19 and 20, most students often or occasionally have the opportunity for stage performance or competition during their study in school, and only 14% of students have no such opportunity. When students are in school, they often have fewer opportunities to play accompaniment in cooperation with instrumental music or vocal music. 43% of students have never had such opportunities. The survey reflects that students lack practical opportunities [19].

### 3.3. Summary of Piano Teaching Problems

#### 3.3.1. The Teaching Mode Lags behind

Generally speaking, in the process of teaching a piano, the students' playing, that is, “returning to class,” is the first part of the teaching process, and the other part is the teacher's evaluation and guidance. This general mode is seen in Figure 2.

However, with the development of the economy and society and the general improvement in national music cultural literacy, especially with the development of quality education in colleges and universities, more students majoring in Musicology in colleges and universities have already had, even a certain level of performance before entering the school. In the past, this effective teaching model for “baiding” students no longer meets the current students' teaching expectations. In the same way, we can know that there must be an obvious gap between students' expectations and teaching effect regardless of any of the traditional above models. This gap is mainly reflected as follows: students cannot express their opinions timely and fully in the teaching process, so that the piano teaching process relies too much on the existing experience and thinking of teachers under the guidance of the established model. This shows that it can undoubtedly be regarded as a waste of teaching resources to some extent [20].

#### 3.3.2. Single Teaching Form

Traditional professional piano teaching adopts the “one-to-one” teaching method. Students learn as teachers teach. This teaching method emphasizes the transmission of knowledge and the learning of skills, and students are in a very passive position. According to the different characteristics of each student and according to the differences in students' piano skill level and knowledge cultivation, the teaching plan in line with the actual situation of students is not formulated; different teaching methods are selected and specific teaching materials are determined for teaching [21]. This single piano teaching mode is often taught by teachers directly, so teachers pay attention to teaching students' playing skills in the teaching process, and it is easy to ignore practical skills and theoretical knowledge. Due to overemphasis on the basic training in performance and ignoring the practical application of piano skills, the performance of impromptu accompaniment and cooperative repertoire is not good. In addition, in the process of teaching each student, teachers need to teach students again and again, which leads to the waste of teachers' energy and equipment resources, and indirectly leads to the decline in teaching quality and restricts the formation of students' creative ability [22].

#### 3.3.3. Lack of Professional Basic and Theoretical Courses

With the vigorous development of colleges and universities in China, China has a large number of music colleges and more colleges and universities with music majors. In these schools, the piano is a basic or compulsory course. However, the source of students majoring in Musicology in colleges and universities is different from that in professional music and art colleges. Most of them have a weak piano foundation before entering school, some have basically never learned piano, and the time of practicing piano in school is also limited. For a long time, the piano courses of music education majors in colleges and universities in China simply copy and imitate the piano performance majors in professional colleges. Blind pursuit of playing skills, while ignoring the cultivation of basic theoretical knowledge of piano, is present. They are not good at guiding students to accurately grasp the most basic and common knowledge and content in piano learning. Students majoring in Musicology in colleges and universities are adults. Their learning purpose is very clear, and they have a strong understanding and thinking ability, perseverance, and acceptance ability [23]. In terms of teaching content, we should strengthen the study of piano theoretical knowledge, guide practice with theory, and need not overemphasize basic skills, otherwise, students will only play a few works when they graduate. At the same time, we should set up courses such as piano teaching methods, systematically teach the basic principles of piano teaching, understand the selection and application of basic piano teaching materials, enable students to master the basic teaching methods of piano learning, and deepen the theory in teaching practice [24].

## 4. Piano Teaching Reform in Colleges and Universities under Diversified Environment

### 4.1. Arming the Traditional Classroom with Piano “Micro Class” Teaching

#### 4.1.1. Relying on “Micro Class” to Realize the “Flipped Classroom” Teaching of Piano in Higher Vocational Colleges

First, optimize the teaching link of “flipped classroom” through the production of “micro class” courseware. By adding professionally designed “micro class” videos to the courseware, constantly optimizing the classroom structure, and penetrating into the teaching tasks and talent training objectives of piano teaching, students can have a more real teaching feeling in the development of piano teaching and give feedback to teachers in time. In this way, we can further strengthen the teaching organizers to improve and break through the weak links in students' piano learning with purpose and method, The second is to form a good interaction of “flipped classroom” through “micro class” resources. In the “flipped classroom” of piano teaching in higher vocational colleges, music teachers should fully mobilize the relationship between students and between students and knowledge through the “micro class” teaching platform, and trigger students' learning enthusiasm through the “micro class” resources with rich content and diversified types. At the same time, teachers can improve the activity of “flipped classroom” through the teaching mode of free discussion, realize the complementary advantages between students through teaching communication and interactive communication, and promote the comprehensive improvement of piano theory and practical skills in higher vocational colleges. In addition, on this basis, the teaching organizer can also arrange the link of reporting the performance, push the piano classroom atmosphere to a climax, and conduct an on-site assessment of students' comprehensive performance through the comprehensive evaluation method of self-evaluation and mutual evaluation to implement the teaching role of “flipped classroom” [25].

#### 4.1.2. Relying on “Micro Class” to Build Piano Education Resource Site

The construction of piano education resource sites in higher vocational colleges can also be continuously completed through “micro course” teaching resources. Through the continuous enrichment of “micro class” teaching resources, we can accumulate the reserves of piano education and teaching resources. Piano teachers in higher vocational colleges should summarize some restrictive factors in the “micro class” classroom teaching, edit it into a “micro class” video suitable for higher vocational students, and then accumulate materials from multiple angles to find targeted and effective solutions so as to promote students to constantly overcome these problems and achieve good learning results. At the same time, piano teachers should make full use of various “micro class” forms to integrate the key and difficult problems and knowledge in piano teaching into the resource site so as to consolidate the professional foundation of students through this form. It can also integrate the rich resources of famous piano players, establish a scientific and systematic network platform, and make full use of the Internet to expand the publicity of high-quality teaching resources so as to benefit teachers at different levels and improve the overall development of piano education level in higher vocational colleges. Due to the short teaching time of “micro lessons,” teachers can give full play to all the teaching skills of “micro lessons.” Through the demonstration of “micro class” video, the database of difficult piano knowledge and skills in higher vocational colleges is established and enriched so as to make a scientific plan for higher vocational students on how to break through these difficulties, master the correct fingering, and gradually form skilled performance skills. Obviously, relying on the “micro course” to build a piano education resource site has expanded the teaching platform and teaching channels for piano teaching in higher vocational colleges, and assisted the development of classroom teaching in a great way. It can not only effectively improve students' ability of independent piano learning but also promote students to constantly find and think about problems in learning, and gradually improve the comprehensive quality and ability of piano theory and practice. At the same time, it has laid a solid foundation for the construction of the overall resource system of music teaching in higher vocational colleges.

#### 4.1.3. Developing Networked Piano Music School-Based Teaching Materials Based on “Micro-Courses”

In comparison, the optimization and integration of piano music network services are more in line with the development of multidisciplinary colleges. Improving the communication of piano music in the school curriculum as a “micro-class” training will make piano instruction in college more colorful and interesting. As a result, colleges and universities can rely on “micro-classroom” courses to create on-campus piano music instructional materials for students. With the new concept of learning networks today, in-school learning materials can be used in conjunction with the realities of student learning to better utilize the educational resources of “micro-class” for improving piano performance goods. The selection of the content of the “micro classes” should be based on the writing and distribution of students' favorite piano music, cognitive skills, and other instructional materials in the school for piano, and support the development of a piano network curriculum in the network. To strengthen the presentation and distribution of this online music.

### 4.2. Making Use of New Media to Create a Networked Piano Learning Environment

#### 4.2.1. Video Network Display of Competitive Student Piano Performance

The first is to build an open competition environment, create an art practice platform for students, allow students show their talents under a relaxed attitude, and be able to choose their favorite piano works for free performance, forming a strong competitive atmosphere. While displaying students' competitive performances on the Internet, different contestants and viewers can interact on the Internet and communicate with each other on piano playing skills and emotional experiences. Obviously, such teaching practice not only exercises students' actual performance ability but also effectively improves students' ability to adjust their psychological quality, as well as their ability to control the stage comprehensively, so as to lay a solid professional foundation for students' future stage performance and teaching. It also plays the role of network teaching and communication. Through the online video competition display of students' piano performance, students can watch the piano performance through the Internet, learn from each other anytime and anywhere, and influence each other, so that the students of higher vocational colleges can promote and improve each other through the online video, and the comprehensive quality of students can be imperceptibly improved.

#### 4.2.2. Introducing the Piano Teaching Habit of Democratic Communication into the Traditional Classroom

First is the principle of capital sharing. Establishing a culture of piano communication in freedom must come first and foremost to ensure free distribution of learning resources. Colleges need to use a vast array of online resources to transform piano concepts into communication concepts of the subject, promoting piano learning to professionals. teaching, and establishing an independent piano.

Second is the principle of liberalization. Based on the research on piano communication media education, colleges should establish free education for teachers and students. With the widespread use of the new media, teachers and students can study for free without time or space constraints. The role of teachers is not just traditional teaching, but being a teacher and facilitator for student learning. In a networked learning environment, students have the freedom to learn piano. This will be a prerequisite for the improvement of piano instruction, which will establish a sense of independence, and will be a new force for deep re-engineering.

### 4.3. Building the Platform of “Admiring Lessons” in Piano Teaching

#### 4.3.1. Construction of “Admiring Lessons” Platform for Piano Teaching in the School

First of all, there is a need to increase investment, improve the effectiveness of the “Mu Angi” piano learning platform in schools, increase the development of the Internet and information technology, and provide maximum capacity and personnel to develop students' piano knowledge and strengthen piano exercises. To train professionals and student representatives to design the Mu Angi platform, we must launch and establish an online student piano training group, build a leadership team to build communication and communication through new media, and increase collaboration and dialogue to lay a good foundation for the development of the “Mu Angi” platform. We must gradually add “Mu class” instructions to the class and carefully create piano music instructional videos to encourage students to watch and learn to improve students' understanding of “Mu class” piano instructions. Therefore, by intensifying the implementation of the college piano “Mu class” instruction, the development of new forms of teaching has increased students' interest in participating and the performing arts on an ongoing basis.

#### 4.3.2. Construction of Interschool Piano Teaching “Mu Class” Platform

The construction of inter-School Piano Teaching “Mu class” platform should fully rely on the campus network to optimize and integrate teaching resources. All kinds of piano teaching platforms should be built through the campus multimedia teaching platform. Through extensive network resources, a new teaching mode is developed for piano students in higher vocational colleges. Piano teachers can put the carefully designed teaching videos on the campus network platform to contribute teaching resources for the students of our class, our school, and brother schools to learn, and also provide rich teaching materials for more teaching colleagues. At the same time, schools can also spontaneously establish network connections, build interactive learning network groups, and achieve the integration of different network piano teaching resources.

## 5. Conclusion

From a variety of sources, teaching piano online will become an integral part of future piano learning. In order to encourage piano students to study on their own, the “professional college” launched a website about piano learning: “Micro Lessons,” which provides detailed guidance according to students' abilities and simultaneously develops piano music courses in the school. “Internet+” organization of training platform for the innovation and rapid development of piano music learning content and materials.

## Figures and Tables

**Figure 1:** Piano teaching for music majors.

**Figure 2:** General mode of curriculum.

**Table 1:** Source of students.

Option	Subtotal	Proportion (%)
City	43	22
Township	87	44
Countryside	66	34

**Table 2:** Did you learn piano when you entered school.

Option	Subtotal	Proportion (%)
Have been studying since I was 10 years old	25	13
Studied for 1–3 years	57	29
Touched a little before the art exam	87	44
Have not learned	27	14

**Table 3:** Your piano playing level at school is/.

Option	Subtotal	Proportion (%)
Cherny 599 degrees	107	55
Cherny 849 degrees	49	25
Cherny 299 degrees	25	13
Above 740 degreesin Cherny	15	7

**Table 4:** Investigation and statistics of students' weekly piano practice time.

Option	Subtotal	Proportion (%)
2–4 hours	63	32
10–5 hours	85	43
More than 10 hours	48	25

**Table 5:** Students' concerns during piano practice.

Option	Subtotal	Proportion (%)
Can I return the class	65	14
Can I play it completely	148	32
Have I mastered the technical essentials	136	29
Is there a musical treatment	114	25

**Table 6:** Does students consult relevant literature and audio-visual materials and learn from them before playing works?

Option	Number of people	Proportion (%)
Often	70	36
Occasionally	104	53
Never	22	11

**Table 7:** Apart from piano solo works, are you exposed to some cooperative works?

Option	Number of people	Proportion (%)
Often	21	11
Occasionally	94	48
Never	81	41

**Table 8:** What do you think of your improvisation ability?

Option	Number of people	Proportion (%)
Can play the piano well	15	8
Can play a little through contact	111	56
Can't play the piano at all	70	36

**Table 9:** Are you interested in piano impromptu accompaniment courses?

Option	Number of people	Proportion (%)
Yes	176	90
No	11	6
Indifferent	9	4

**Table 10:** Will the school provide enough piano for practice?

Option	Subtotal	Proportion (%)
Yes	93	47
No	103	53

**Table 11:** Whether the school library has enough literature and audio-visual materials?

Option	Subtotal	Proportion (%)
Yes	77	39
No	119	61

**Table 12:** Whether teachers involve relevant music-theoretical knowledge in piano teaching?

Option	Subtotal	Proportion (%)
Often	75	38
Occasionally	102	52
Never	19	10

**Table 13:** Does the teacher discuss the daily piano practice methods with you in piano teaching?

Option	Subtotal	Proportion (%)
Often	61	31
Occasionally	104	53
Never	31	16

**Table 14:** Application of teachers in piano teaching.

Option	Subtotal	Proportion (%)
Technical training	34	17
Musical feeling	23	12
Combination of the two	139	71

**Table 15:** Teachers pay more attention to piano teaching.

Option	Subtotal	Proportion (%)
Piano playing ability	139	71
Sight reading ability	22	11
Impromptu accompaniment ability	8	4
Cooperation ability	27	14

**Table 16:** Teachers' common use in piano teaching (multiple choices).

Option	Subtotal	Proportion (%)
Teaching method	129	22
Discussion method	46	8
Model method	155	26
Drill method	107	18
Conversation method	54	10
Edification method	24	4
Inquiry method	39	6
Other	39	6

**Table 17:** What is the teaching form of your piano lessons?

Option	Subtotal	Proportion (%)
Individual course	78	40
Group course	83	42
Collective course	34	18

**Table 18:** Does your school organize lectures, concerts, and other academic exchange activities?

Option	Subtotal	Proportion (%)
Often	91	46
Occasionally	88	45
Never	17	9

**Table 19:** Are there any opportunities for stage performances (or competitions) during school study?

Option	Subtotal	Proportion (%)
Often	71	36
Occasionally	98	50
Never	27	14

**Table 20:** During school study, are there opportunities for other instrumental or vocal accompaniment?

Option	Subtotal	Proportion (%)
Often	30	15
Occasionally	82	42
Never	84	43

## Data Availability

The labeled data set used to support the findings of this study is available from the corresponding author upon request.
